# Clinical Effect of Flexible Ureteroscope and Laparoscope in the Treatment of Parapelvic Cyst

**DOI:** 10.1155/2022/5718923

**Published:** 2022-10-04

**Authors:** Ruipeng Tang, Jie Yang, Li Wan, Zhengrong Yang

**Affiliations:** ^1^General Hospital of Pangang Group, China; ^2^Huidong County People's Hospital, China

## Abstract

**Objective:**

Comparing the clinical effect of flexible ureteroscope and laparoscope in the treatment of parapelvic cyst.

**Method:**

A total of 82 patients with parapelvic cyst who underwent surgical treatment in our hospital from May 2019 to May 2020 were selected. Patients were randomly divided into a control group and an observation group; the control group underwent laparoscopic parapelvic cyst topical decompression; the observation group underwent transurethral flexible ureteroscope holmium laser incision and drainage of parapelvic cyst. The intraoperative (operative time, intraoperative blood loss, and ventilation time), postoperative (time of getting out of bed, pain score, and length of hospital stay), and recurrence were compared between the two groups.

**Results:**

(1) The operative time and intraoperative blood loss in the observation group were significantly better than those in the control group (*P* < 0.05), while the ventilation time had no significant difference (*P* > 0.05). (2) The pain score and length of hospital stay in the observation group were better than those in the control group (*P* < 0.05). There was no significant difference in the time of getting out of bed (*P* > 0.05). (3) There was no serious infection or bleeding in either group. The observation group had no recurrence, and the postoperative recurrence rate was 0. There were 11 cases of recurrence in the control group, and the postoperative recurrence rate was 26.83%. The postoperative recurrence rate of the observation group was significantly lower than that of the control group, with statistical significance (*χ*^2^ = 4.604, *P* < 0.05).

**Conclusion:**

Flexible ureteroscope for the treatment of parapelvic cyst could effectively reduce the operative time, intraoperative blood loss, and pain; in addition, the postoperative recovery was fast and the recurrence is rare, which was worth popularizing.

## 1. Introduction

Pararenal cyst is developed from simple renal cyst. The cyst wall is covered by a thin layer of fibrous tissue with a layer of flat epithelium, containing straw yellow clear liquid. A few cysts contain bloody liquid. After infection, the wall can be thickened, containing viscous liquid [1]. Patients with pain symptoms or great psychological effects or cyst diameter > 4 cm or < 4 cm need active surgical treatment to avoid kidney damage [2, 3]. Most renal cyst is located in the renal surface, or inside renal parenchyma, and has partial renal cyst to be located inside the renal sinus; the relation with renal pelvis is relatively close; this kind is called renal pelvis side cyst [4]. It is often accompanied by low back pain, hydronephrosis, hematuria, and high blood pressure, combined with kidney stones, infection, and so on [5, 6]. Parapelvic cysts have a greater impact on the function of the kidneys and the body. Due to the particularity of their onset location, they are often confused with other lesions in the renal pelvis area [7]. Laparoscopic decompression of parapelvic cyst is the preferred method for the treatment of parapelvic cyst. However, due to the special location of the parapelvic cyst near the renal pedicle, laparoscopic surgery is risky [8]. The risks of laparoscopic pararenal cyst surgery mainly include the following aspects: (1) incision infection. Because the laparoscopic incision requires the placement of an operating frame, the incision is prone to infection and delayed healing. (2) Renal hemorrhage, which is often seen when the cyst wall is removed and the renal parenchyma is damaged too much. (3) Cyst recurrence. Cysts have a certain recurrence rate, which is related to too little excision of the swelling wall and too deep swelling location [9, 10]. Studies have shown that intraureteral incision and drainage for cysts under flexible ureteroscope is safe and has definite short-term efficacy, but the long-term efficacy and complications remain unclear [11, 12]. 82 patients with parapelvic were selected as the research subjects. The intraoperative (operative time, intraoperative blood loss, and ventilation time), postoperative (time of getting out of bed, pain score, and length of hospital stay), and recurrence were compared between the two groups.

## 2. Materials and Methods

### 2.1. General Information

82 patients with parapelvic cyst who underwent surgical treatment from May 2019 to May 2020 were selected as the research subjects. There were 41 cases in each group. The control group had 20 female patients and 21 male patients. The average age was 57.65 ± 5.12 years from 43 to 75 years old. The cyst diameter was 3.32~6.12 cm, with an average of 4.86 ± 0.79 cm, cyst location: bilateral 12 cases, left 13 cases, and right 16 cases. In the observation group, there were 19 females and 22 males, age 42~75 years old, average 57.61 ± 5.03 years old. The diameter of the cyst was 3.12~6.25 cm, and the average was 5.13 ± 0.79 cm, cyst location: bilateral 12 cases, left 12 cases, and right 17 cases. There was no significant difference in the above general data between the two groups (*P* > 0.05); it was comparable. This study was carried out with the approval of the Ethics Committee of our hospital.

1. Inclusion criteria: (1) all patients were clinically diagnosed as having parapelvic cyst; (2) single parapelvic cyst, > 4 cm in diameter, or associated with low back pain; and (3) signed an informed consent
2. Exclusion criteria: (1) severe disturbance of consciousness; (2) severe hepatic and renal dysfunction; and (3) patients who were not eligible for this study

General information is shown in Table 1.

### 2.2. Methods

Laparoscopic ureterolithotomy is applicable to the treatment of upper and middle ureteral calculi. First, the passage of laparoscopy should be established, which is generally composed of 2-3 operating holes of a lens hole. Then, the ureter should be free, and the ureters at both ends of the stone should be fully free, and then, the urinary catheter should be cut to remove the stone [13]. The control group underwent laparoscopic parapelvic cyst topical decompression; general anesthesia for endotracheal intubation (the purpose of endotracheal intubation is to administer anesthesia, and its main risk is anesthesia risk, which is divided into poor anesthesia effect to patient pain or shock. The operation flow of tracheal intubation anesthesia is shown in Figure 1) was performed. The control group was placed in 45° oblique position on the healthy side, 1 cm of skin was cut under the navel, and the abdominal wall was lifted with cloth forceps on both sides. The Veress needle (the Veress needle is composed of Veress needle outer sheath, Veress needle inner core, ventilation switch, and other components. The outer sheath of the Veress needle is generally 2 mm in diameter and 80 mm, 120 mm, and 150 mm in length. It is composed of a sharp needle sheath and a blunt needle core. The front end of the needle core is round and hollow and has side holes, which can be used for gas injection, water injection, and suction through the needle core. The Veress needle is a clinical medical instrument used for abdominal puncture) was used to puncture into the abdominal cavity, and the pneumoperitoneal machine was given to boost the pressure; then, a 10 mm Trocar was implanted. Under the guidance of laparoscopy, 10 mm Trocar and 5 mm Trocar were implanted in the midpoint of the line between umbilicus and xiphoid process and under the costal front axillary line, respectively. Separate the colon to the healthy side, and open the lateral peritoneum along the paracolic sulcus, as well as the hepatocolonic ligament or the splenocolonic ligament, the perirenal fascia, and fat sac were opened at the renal sinus to separate and expose the parapelvic cyst, avoiding damage to renal vessels and renal pelvis [14]. Lift the cyst wall, cut the cyst wall, remove the cyst wall as much as possible, and finally use the electrocoagulation hook to electrocoagulate the edge. Drainage tubes were placed around the kidney, and the incision was closed.

The method of holmium laser cutting under ureteroscopy is to use a flexible ureteroscope and then enter the ureter after passing through the urethra and bladder. The stones in the patient's body are broken and removed with a holmium laser. The advantage of this method is that it uses the natural urinary tract of the human body, so it does not make any incision on the body, which belongs to a relatively pure endoscopic minimally invasive surgery. Compared with laparoscopic ureterolithotomy, it has great advantages, such as less trauma, wide applicability, and rapid recovery [15]. The observation group underwent transurethral flexible ureteroscope holmium laser incision and drainage of parapelvic cyst; general anesthesia was administered; they were placed in a lithotomy position; a hard ureteroscope was inserted into the renal pelvis; the ureter is inspected; indwelling a hydrophilic guide wire into the renal pelvis, the flexible ureteroscope dilated sheath was placed along the guide wire to the ureteropelvic junction; and the inner core was removed. An electronic flexible ureteroscope was inserted into the renal pelvis to examine each calyx and renal pelvis in turn. Identify the location of the cyst (blue translucent projection or gray projection of the renal pelvis and calyces mucosa; if the exploration was difficult, intraoperative ultrasound could be used to locate the cyst). The thinnest part of the cyst wall was cut radially with 200 *μ*m holmium laser fiber (25~30 Hz, 0.8~1.0 J), and the window diameter was 1~2 cm, so that the cyst cavity was completely communicated with the renal pelvis, and whether there was space occupying at the bottom of the cyst was examined [11]. If renal calculi were complicated, the patients were first treated with 200 *μ*m holmium laser lithotripsy; then, the calculi were removed with a stone basket, and then, the cyst was incised. Indwelling F7 double J tubes were fully drained in the cyst lumen, and the tubes were removed one month after operation.

### 2.3. Observational Index

Operative time, intraoperative blood loss, and ventilation time are the important indicators considered in the operation of pararenal cyst. Ventilation is the so-called exhaust. Generally speaking, it means farting. It means that the intestines and stomach recover peristalsis and you can eat. “Ventilation time” refers to the period from the operation of pararenal cyst to intestinal ventilation. Pain was scored using visual analogue scoring method, with a total score of 10. The more severe the pain, the higher the score.

### 2.4. Statistical Methods

The statistical software SPSS23.0 was used for data processing. The measurement data were compared by *t* test, and the enumeration data were compared by *χ*^2^ test.

## 3. Results

### 3.1. Intraoperative Result

The operative time and intraoperative blood loss in the observation group were significantly better than those in the control group (*P* < 0.05), while the ventilation time had no significant difference (*P* > 0.05). Intraoperative result is shown in Table 2.

### 3.2. Postoperative Result

The pain score and length of hospital stay in the observation group were better than those in the control group (*P* < 0.05). There was no significant difference in the time of getting out of bed (*P* > 0.05). Postoperative result is shown in Table 3.

### 3.3. Result of Recurrence

There was no serious infection or bleeding in either group. The observation group had no recurrence, and the postoperative recurrence rate was 0. There were 11 cases of recurrence in the control group, and the postoperative recurrence rate was 26.83%.

## 4. Discussion

Parapelvic cyst is a kind of more serious urological disease, mainly developed from simple renal cyst, which has serious harm to the health of patients. Its clinical treatment is generally based on surgery; there are many ways; the surgical effect is also different [16]. There is no medicine or traditional Chinese medicine method that can eliminate or reduce the pararenal cyst. Surgical resection is adopted. The common surgical resection methods are as follows: (1) laparoscopic cyst resection; (2) cyst decapitation decompression or cyst resection; (3) puncture and aspirate cyst fluid and inject sclerosing agent under the positioning of B-ultrasound; and (4) unilateral parapelvic cysts can be treated by retroperitoneal approach, and bilateral cysts can be treated by intraperitoneal approach at the same time [17]. Parapelvic cyst refers to the cyst occurring near the renal pelvis and is a rare type of renal cystic diseases, accounting for 1%~3% of renal cystic diseases [18]. Because the anatomical location of the parapelvic cyst is close to the renal hilum, it often oppresses renal blood vessels, collecting system and lymphatic vessels and causing pain, hematuria, hydronephrosis, infection, and so on; severe cases can lead to glomerulonephritis, renal vascular hypertension, and even renal failure, so more aggressive treatment measures should be taken once found [19, 20]. Due to the particularity of the site of occurrence, parapelvis cysts are more harmful to people than cysts in renal parenchyma or renal surface. Surgical treatment is recommended when clinical symptoms appear [21, 22]. Due to the location of the parapelvic cyst adjacent to the renal pelvis, renal hilum, and other structures, percutaneous renal cyst puncture sclerosis has the risk of damage to the renal pelvis or renal hilum structure, and urinary fistula or renal vascular rupture and bleeding easily occur [23]. Ureteroscopy can completely observe more than 96% of the intrarenal collecting system and treat it, especially the upper ureteral calculi. When doctors perform surgery, the stones at the upper end of the ureter may move into the kidney. The ureteroscopy can find the kidney stones or the stones that move up by bending the front end and treat them, so the treatment scope of ureteroscopy is broader [24]. Open surgery has larger trauma, longer recovery time, and more postoperative complications. Therefore, for the treatment of pararenal cyst, clinicians use minimally invasive surgery such as flexible ureteroscopy and laparoscopy rather than open surgery. The advantages of laparoscopy and flexible ureteroscope are that the surgical wound is small (usually only three channels), the operation is safe, and the postoperative recovery time of patients is short [25]. The treatment of parapelvic cyst by a flexible ureteroscope has the advantages of short operation time, small surgical trauma, less intraoperative bleeding, quick postoperative recovery, short postoperative hospitalization, and so on. Most hospitals in China choose laparoscopic surgery as the first choice for treatment [26, 27]. Internal incision and drainage of parapelvic cyst under a flexible ureteroscope is a more natural lumen approach, and there is basically no blind area, so that the location of the cyst can be more accurate [28].

This study showed that (1) the operative time and intraoperative blood loss in the observation group were significantly better than those in the control group (*P* < 0.05), while the ventilation time had no significant difference (*P* > 0.05); (2) the pain score and length of hospital stay in the observation group were better than those in the control group (*P* < 0.05). There was no significant difference in the time of getting out of bed (*P* > 0.05). (3) There was no serious infection or bleeding in either group. The observation group had no recurrence, and the postoperative recurrence rate was 0. There were 11 cases of recurrence in the control group, and the postoperative recurrence rate was 26.83%.

## 5. Conclusion

In conclusion, there is no medicine or other nonsurgical means to eliminate or reduce the pararenal cyst. Patients and urologists need to choose the appropriate surgical method according to the individual situation of patients. A flexible ureteroscope for the treatment of parapelvic cyst could effectively reduce the operative time, intraoperative blood loss, and pain; in addition, the postoperative recovery was fast and the recurrence is rare, which was worth popularizing.

## Figures and Tables

**Figure 1:** The operation flow of tracheal intubation anesthesia.

**Table 1:** General information.

Groups	Control group	Observation group	*P*
Cases	41	41	
Age	57.65 ± 5.12	57.61 ± 5.03	>0.05
Gender (male/female)	21/20	22/19	>0.05
Cyst diameter (cm)	4.86 ± 0.79	5.13 ± 0.79	>0.05
Cyst location (bilateral/left/right)	12/13/16	12/12/17	>0.05

**Table 2:** Intraoperative result.

Groups	Cases	Operative time	Intraoperative blood loss	Ventilation time
Control group	41	65.78 ± 16.32	100.34 ± 16.33	1.44 ± 0.58
Observation group	41	40.36 ± 14.57	18.32 ± 7.21	1.04 ± 0.49
*P*		<0.05	<0.05	>0.05

**Table 3:** Postoperative result.

Groups	Cases	Pain score	Time of getting out of bed	Length of hospital stay
Control group	41	4.91 ± 1.65	1.38 ± 0.29	5.18 ± 1.03
Observation group	41	3.48 ± 1.52	1.21 ± 0.24	4.21 ± 1.02
*t*		2.064	3.104	2.101
*P*		<0.05	>0.05	<0.05

## Data Availability

The data used to support the findings of this study are included within the article.
